The article "Neurobehavioral Effects of Restricted and Unpredictable Environmental Enrichment in Rats" was published in 2020. Journal: Front Pharmacol.

# Neurobehavioral Effects of Restricted and Unpredictable Environmental Enrichment in Rats

**DOI:** 10.3389/fphar.2020.00674

**Published:** 2020-05-12

**Authors:** Mijail Rojas-Carvajal, Andrey Sequeira-Cordero, Juan C. Brenes

**Affiliations:** ^1^ Neuroscience Research Center, University of Costa Rica, San Pedro, Costa Rica; ^2^ Institute for Psychological Research, University of Costa Rica, San Pedro, Costa Rica; ^3^ Institute for Health Research, University of Costa Rica, San Pedro, Costa Rica

**Keywords:** environmental enrichment, neural plasticity, motivation, ultrasonic vocalizations, grooming, learning, emotion, reward

## Abstract

To study how motivational factors modulate experience-dependent neurobehavioral plasticity, we modify a protocol of environmental enrichment (EE) in rats. We assumed that the benefits derived from EE might vary according to the level of incentive salience attributed to it. To enhance the rewarding properties of EE, access to the EE cage varied randomly from 2 to 48 h for 30 days (REE). The REE group was enriched only 50% of the time and was compared to standard housing and continuous EE (CEE) groups. As behavioral readout, we analyzed the spontaneous activity and the ultrasonic vocalizations (USVs) within the EE cage weekly, and in the open field test at the end of the experiment. In the cage, REE increased the utilization of materials, physical activity, and the rate of appetitive USVs. In the OF, the CEE-induced enhancements in novelty habituation and social signaling were equaled by the REE. At the neural level, we measured the expression of genes related to neural plasticity and epigenetic regulations in different brain regions. In the dorsal striatum and hippocampus, REE upregulated the expression of the brain-derived neurotrophic factor, its tropomyosin kinase B receptor, and the DNA methyltransferase 3A. Altogether, our results suggest that the higher activity within the cage and the augmented incentive motivation provoked by the REE boosted its neurobehavioral effects equaling or surpassing those observed in the CEE condition. As constant exposures to treatments or stimulating environments are virtually impossible for humans, restricted EE protocols would have greater translational value than traditional ones.

## Introduction

Knowing about how animals react to different environmental conditions would contribute to explaining why environmental stimulation in humans (e.g., physical and psychological therapies, exercise, and preventive or palliative treatments) benefits some subjects but not others, a crucial enigma about the complex relationship between experience and neurobehavioral plasticity. The positive impact of environmental stimulation in humans may rely upon attributions and expectations about their own performance and the putative benefits derived from the treatments (Benedetti et al., 2004; Knutson et al., 2005; Scott et al., 2007), suggesting that motivational factors are key modulators of the entire effect. However, the study of how motivation contributes to the benefits of environmental stimulation has received little attention in health sciences, and even less in preclinical research.

To study the likely role of motivation in the regulation of experience-dependent plasticity on brain and behavior, we first redesigned a protocol of environmental enrichment (EE) in rats and then assessed its effects on different behavioral domains and the expression of genes related with neural plasticity (**Figure 1**; **Table 1**). EE consists of exposing laboratory rodents to physical and social stimulation higher than the one received in standard laboratory housing (Rosenzweig and Bennett, 1996; Crofton et al., 2015), with physical exercise, social activity, and the exposure to complex and constantly changing stimuli as the triad of enriching factors affecting behavior and brain function (Bekinschtein et al., 2011; Crofton et al., 2015; Brenes et al., 2016; Ohline and Abraham, 2019). We assumed, therefore, that the benefits derived from EE may be determined by motivational factors related to how much animals attribute incentive salience to such stimulations. The motivational value of an appetitive stimulus can be potentiated through unpredictable presentations (Anselme et al., 2013; Schultz, 2016; Kreisler et al., 2018). Thus, to enhance the rewarding properties of the EE, we developed a protocol in which access to the EE cage was restricted to specific durations ranging from 2 to 48 h unpredictably for 30 days. Rats in the restricted and unpredictable EE (REE) condition were compared with rats exposed continuously to EE (CEE), with REE animals remaining only 50% of the total time in the EE cage throughout the housing period (**Figures 1C, D**). Contrary to most EE protocols described so far, our EE protocols consisted of a selection of natural, previously screened stimuli, which were classified into broad categories according to the function they may serve (e.g., dens and hideouts, sensorimotor and physical stimuli, nesting and chewing materials, and highly palatable foods). During the non-EE period, the REE rats were housed five in standard housing (SH) cages. Thus, two control groups were used: one with five rats per cage (SH5) to match the housing of REE rats, and a group with two rats per cage (SH2) with less social contact, which served as a control group of all other conditions.

**Figure 1:** Housing conditions and experimental design. **(A)** Transparent, polycarbonate cage (56 cm × 35 cm × 20 cm) filled with ~5 L of bedding for standard housing (SH). **(B)** Custom-made (135 cm × 68 cm × 110 cm), environmental enrichment (EE) cage surrounded by wire-mesh walls consisting of four stainless steel levels interconnected by metal and wooden stairs. The cage contained dens, hideouts, nesting and chewing materials, different objects for sensorimotor stimulation, feeders, and two bottles of water (for details see **Table 1**). The first floor was always covered with bedding and had a sandbox. No running wheels were used. **(C)** Distribution of groups (n = 10 rats per group). SH2: pair-housed rats in SH cages; SH5: five rats per cage in SH cages; CEE: ten rats per cage exposed continuously to EE throughout the 30-days protocol (~720 h), except during bed changes (30 min) when rats were housed in groups of five in SH cages; REE: 10 rats per cage with restricted and unpredictable access to the EE cage during ~360 h (50% of the CEE total time). For the REE rats, the time in the cage was equally distributed between the light and dark cycle, with exposures to the EE cage ranging randomly from 2 to 48 h. During the non-EE periods, these animals were also housed in groups of five in SH cages. CEE and REE rats were housed in independent EE cages. In order to control the increased handling experienced by REE rats, both SH groups and CEE rats were also handled each time REE rats were put in and out the EE cage: while SH2 and SH5 animals were relocated into new cages, CEE rats were group-housed in SH cages (fiveper cage) during 5 min and then returned into the EE cage. **(D)** Experimental design. Housing conditions started at postnatal (PND) 29 and continued throughout 30 days. In experiment 1, behavioral activity and USVs within the EE cage were measured once a week (Wk) after bed changes. At PND 59, animals were tested on four, one-day apart open-field (OF) tests for 15 min. In experiment 2, SH5, CEE, and REE groups were included (n = 10 rats per group) and animals were housed exactly as in experiment 1. No behavioral assessments were carried out to these animals. At PND 59, rats were euthanized, and their brain tissues were collected for mRNA quantification of BDNF, TrkB, CREB, p250GAP, and DNMT3A genes on the hippocampus, the dorsal striatum, and the nucleus accumbens.

**Table 1:** A detailed description of the items used for environmental enrichment.

Use and purpose	Item	Material	Dimensions	N	Company	Behavior elicited
Dens and hideouts	Ball nest	Grass	Diameter: 22.86 cm	2	Prevue Hendryx^®^	Accumulation Nest building Hiding Chewing Jumping Chasing
	Cross tube	Grass	35.56 × 35.56 cm; diameter: 10.8 cm	2	Prevue Hendryx^®^	
	Bird nest	Grass	Height: 29 cm; diameter: 14 cm	2	Prevue Pet Products^®^	
	Squared cross tube	Cedar wood	20 × 20 × 10 cm	2	Custom made	
	Squared tube	Cedar wood	20 × 10 × 10 cm	2	Custom made	
	Boxes	Paperboard	30 × 20 × 10 cm	1	Custom made	
	Round tubes	Bamboo	22 cm; diameter: ~9 cm	2	Custom made	
	Rodent houses	Pine wood	26 × 35.36 × 21 cm	2	Kaaytee^®^	
	Small round tubes	Paperboard	17 × 4.5 cm	2	Tork^®^ (paperboard residue of paper towels)	
Sensorimotor and physical stimuli	Stairs	Pinewood	88 x 10 cm	2	Custom made	Climbing Jumping Chewing Littering Play Digging/burring feces
	Square blocks	Raw wood	7.5 × 7.5. × 7.5 cm	4	Custom made	
	Round blocks	Cedar wood	Diameter:12 cm; height: 4 cm	4	Custom made	
	Boulders	Rock	Variable size	4–6	Local supplier	
	Woven ball	Natural wood fiber	~15 cm	2	Ware manufacturing^®^	
	Rope^1^	Polypropylene	100 cm	1	Local supplier	
	Sandbox^1^	Steel	27.5 × 26.5 × 4 cm	1	Custom made	
	Sand^1^	Sand	–	~1 L	Purina^®^	
Nesting and chewing materials	Tissues	Paper, cotton	Standard size	8	Kleenex^®^	Chewing Dragging Nest building
	Bedding^1^	Pinewood	~3 × 3 cm	~10 L	Local supplier	
	Hey	Natural hey	Variable	~1 L	Local supplier	
	Hard paper^1^	Kraft paper	124 × 60 cm	1	Local supplier	
	Wood sticks	Wood	~15 × 0.5 cm	8–10	Local supplier	
Highly palatable food^2^	Sunflower seeds	Natural dry seed	Variable	400 ml	Local supplier	Foraging Chewing Climbing Incentive motivation
	Cheerios^®^	Oat, corn	Variable	400 ml	General Mills^®^	

^1^These objects were always included in all the configurations of the cage.

^2^During the first week of housing, the small feeders filled with highly palatable foods were placed in the first level of the EE cage. In the following weeks, they were hung up randomly on different locations of the cage walls and relocated during bed changes.

Experiment 1 consisted of two phases. In the first phase, we evaluated the psychomotor and motivational responses toward the EE cage and compared the two EE protocols in that regard. Accordingly, we assessed once a week the exploratory activity, the use of materials, the eating-related behaviors, the social interactions, and the ultrasonic vocalizations (USVs) within the EE cages (**Figure 4C**). USVs are socio-affective signals serving distinct communicative functions in the rat. The so-called 22-kHz calls are emitted as alarm signals in aversive situations, whereas 50-kHz calls consist of many different subtypes appearing in social and non-social situations of neutral or positive affective valence (Brudzynski, 2013; Simola and Brudzynski, 2018). In the second phase, we analyzed the spontaneous activity and the USVs emitted in the open field (OF) after the 30-days housing period, to identify the behavioral effects of our EE protocols, which were compared between each other and with the SH groups. The OF was selected as it is one of the most consistent behavioral paradigms to detect the effects of EE (Elliott and Grunberg, 2005; Brenes Sáenz et al., 2006; Sampedro-Piquero et al., 2018). Besides measuring locomotion and rearing, we performed a detailed analysis of the different grooming subtypes as they may be informative of particular learning and emotional processes (e.g., novelty habituation and emotional de-arousal) and because they are very responsive to EE (**Figure 2**) (Spruijt et al., 1992; Brenes et al., 2009; Rojas-Carvajal et al., 2018). We also measured in the OF the spontaneous 50-kHz calls elicited when rats are transiently separated from conspecifics (**Figure 7**, lower right panel) (Wöhr et al., 2008; Natusch and Schwarting, 2010). These USVs are considered as an index of prosocial behavior co-occurring during risk assessment, which can be modulated by social and physical EE and are responsive to repeated testing and stress (Schwarting et al., 2007; Wöhr et al., 2008; Brenes et al., 2016, Rojas-Carvajal and Brenes, submitted).

**Figure 2:** Topographical and theoretical analysis of grooming. To understand why a non-exploratory, self-oriented behavior is displayed in the context of unconditioned anxiety tests, such as the OF, we developed a classification considering the kinetics, the anatomical distribution, and the complexity of grooming strokes (Brenes et al., 2009; Rojas-Carvajal et al., 2018; Rojas-Carvajal and Brenes, submitted). Based on its anatomical distribution, grooming was classified as cephalic (1–3), caudal (4), and sequential (1–4). Based on its motor complexity, each anatomical category could also include variations as follows: cephalic (1–3 + 5b, 6), caudal (4 + 5a, 6) and sequential (1–4 + 5a, 5b, 6). Regarding the kinetics, the colored arrow represents the theoretical association between grooming subtypes and defensiveness over time. The red-to-green fading indicates the transition from high defensive arousal to low defensive arousal, with cephalic subtypes appearing at the beginning of testing when exploratory and risk-assessment behaviors are prominent (Brenes et al., 2009; Rojas-Carvajal et al., 2018). With time, sequential grooming with variations gradually appears. As complex and intricate grooming sequences seem to compromise the prompt responses to any oncoming threat, it supposes that rats are now disengaged from displaying defensive responses. Thus, we interpreted the appearance of those subtypes as markers of habituation learning and emotional de-arousal (Brenes et al., 2009; Rojas-Carvajal et al., 2018). Black arrows represent the most common transition between the grooming sequences.

In experiment 2, we analyzed the effects of our EE protocols on the expression of genes involved in neural plasticity. We focused on genes related to the signaling pathway of the brain-derived neurotrophic factor (BDNF) through its tropomyosin kinase B receptor (TrkB). Thus, we also measured the expression of the transcription factor cAMP response element-binding (CREB), which not only belongs to the BDNF/TrkB pathway but also regulates the expression of hundreds of genes, including BDNF (Carlezon et al., 2005; Yu and Rasenick, 2012). The expression of the Rho GTPase activating protein 32 (ARHGAP32, also known as p250GAP) was also analyzed as it is involved in structural plasticity by regulating the molecular changes associated with cytoskeleton remodeling (Nakazawa et al., 2003; Marler et al., 2014). Finally, we measured the expression of the DNA methyltransferase 3A (DNMT3A), as it is responsible for *de novo*-type DNA methylation and for establishing and maintaining proper DNA methylation patterns, which are presumably relevant for neural plasticity at certain genomic loci in postmitotic neurons (Griñan-Ferré et al., 2016; Zhang et al., 2018). These mRNA analyses were performed in SH5, REE, and CEE rats that were not submitted to behavioral assessment. We extracted the nucleus accumbens, dorsal striatum, and hippocampus because 1) they are all involved in different phases of the motivational processes (e.g., attribution of incentive salience, the transition from motivation to action, and contextual encoding of reward cues) (Williams and Undieh, 2010; Anselme et al., 2013; Schultz, 2016); 2) they play a pivotal role on learning and memory (e.g., associative, procedural, and episodic/spatial memory) (Richard et al., 2013; Lisman et al., 2017); and 3) the EE-induced physiological and cellular effects have been well identified in those regions and especially in hippocampus (Bezard et al., 2003; Brenes et al., 2008; Brenes and Fornaguera, 2008; Tipyasang et al., 2014; Brenes et al., 2016; Grimm et al., 2018; Scala et al., 2018; Ohline and Abraham, 2019).

## Materials and Methods

### Subjects

Seventy male Wistar rats were transported to our colony room from LEBi facilities (University of Costa Rica, San José) at postnatal day (PND) 22 ( ± 1). Upon arrival, animals were tail-marked, weighted, and housed with their littermates in a 12:12 light-dark schedule (lights on at 6:00 h), temperature of 22.3°C ( ± 4.5°C), and relative humidity of 71.5% with 10 air cycles/hour. Food and water were provided *ad libitum* and refilled twice per week during bed changes. In experiment 1, the 40 rats were screened in the cage test (CT) as previously reported (Pereira et al., 2014; Brenes et al., 2016). Briefly, the CT consisted of placing a rat individually in a transparent polycarbonate cage (42 × 26.5 × 15 cm) filled with fresh bedding and illuminated at ~10 lumens, where locomotion, rearing, total grooming, and total 50-kHz USVs were measured for 5 min (see below for details). We left only one day of acclimatization between arrival and the CT because the experience of being moved from one cage to another and then returned back to the home cage constitutes a quite standard procedure in any lab, and because after the 5-min test rats remained undisturbed for four days, which can be considered a continuation of the acclimatization period. The groups' allocation procedure consisted of assigning semi-randomly the rats to the experimental groups (n = 10/group) based on body weight, litter of origin, behavioral activity, and USVs in the CT (**Figures 1C, D**), so that the inter-subject variability was equally distributed within the groups, and no subjects were excluded from the sample. In experiment 2 (30 rats), only body weight and the litter of origin were used for group allocation (**Figure 1D**). Housing conditions started at PND 29 in both experiments. All experimental procedures were done according to the guidelines of the Costa Rican Ministry of Science and Technology for the Care and Use of Laboratory Animals and were approved by the Institutional Committee for Animal Care and Use of the University of Costa Rica (CICUA-161-16).

### Housing Conditions

A modified version of our EE protocol was implemented (Brenes Sáenz et al., 2006; Brenes et al., 2009; Mora-Gallegos et al., 2015; Brenes et al., 2016; Rojas-Carvajal et al., 2018). To alleviate the stress of captivity, satisfy some of the ethological needs of the animals, and elicit species-specific behaviors, the proper stimuli should be provided (Olsson and Dahlborn, 2002; Swaisgood, 2007; Tarou and Bashaw, 2007). With this in mind, we adopted a rather naturalistic approach by replacing plastic objects with natural items to the largest extent possible (**Figure 1B**). Based on our previous protocol (Brenes et al., 2016) and pilot studies, we selected several items (see **Table 1**) which were supposed to serve a specific purpose classified into four broad categories: dens and hideouts, sensorimotor and physical stimuli, nesting and chewing materials, and highly palatable foods. Within each category, different items were included. A fixed number of objects per category were distributed into the cage on each configuration, which varied systematically twice per week during bed changes to avoid item repetitions within the same week (**Table 1**). Those objects that always remained in the cage were also rearranged (**Table 1**).

### Kinetics of Spontaneous Activity Within the EE Cage

Once a week after bed changes, behavioral activity and USVs inside the EE cages were scored for 10 min. One camera (GoPro Hero3, USA) was located at the frontal door (90 cm height) for monitoring the overall activity inside the cage. A second camera was located on the cage floor to monitor the activity at the lower levels. Five weekly sessions were recorded on the same days (between 7 and 9 am), starting with a baseline taken the first day of EE. The following behaviors were manually scored in segments of 10 s: running, climbing, jumping, rough-and-tumble, chasing, material accumulation, moving objects, ripping objects or materials, foraging, eating, sniffing, and stretched-attempt posture. For USVs recordings, a microphone hung up from the center of the cage's ceiling at 40 cm above the first floor.

### OF Test

Four rats, one from each group, were tested simultaneously on black Formica, square-wooden chambers (55 cm × 55 cm × 40 cm) located in independent rooms illuminated with white dimmed light (10 ± 1 lumens). Animals were individually placed in the middle of the arena and tested for 15 min. Afterward, the apparatuses were cleansed with ethanol (70%). Behaviors were video recorded (cameras at 80 cm height; GoPro Hero3-4, USA) for offline analysis. Locomotion was automatically scored using the video tracking system Any-Maze (version 5.1, Stoelting Co., Wood Dale, IL, USA) and reported as distance traveled in meters. The frequency of rearing and the duration of grooming were manually scored by trained observers (> 90% inter-observer reliability) using Solomon Coder free software (version 17.03.22; https://solomoncoder.com/download.php). Solomon Coder data was extracted using custom-made macros of Microsoft Office Excel. Rearing consisted of a bipedal posture (> 45° from the floor) where the animal extends its head upwards, executing a series of lateral movements using vibrissae to sense the surroundings. Positions <45° were excluded by being regarded as incomplete postures. We developed a grooming classification system based on its anatomical distribution and its levels of motor complexity (Rojas-Carvajal and Brenes, submitted). Based on its anatomical distribution, we classified grooming into three categories: cephalic (**Figures 2.1–3**: hand rubbing, face washing, unilateral and bilateral strokes), caudal (**Figure 2.4**: body liking and/or anus-genital licking), and sequential (**Figures 2.1–4**: chained events of cephalic and caudal grooming). Regarding grooming complexity, we observed that rats could use the hind paws to perform grooming sequences within each of the previous anatomical categories resulting in six possible grooming subtypes (**Figure 2**). When grooming was interrupted by locomotion (i.e., full displacement by using the four paws) or by any other behavior for >8 s, separated events were counted. If a rearing occurred within a grooming event, its time was discounted from the total grooming duration. Micro grooming (<1 s) events were also counted, but isolated scratching events were discarded (**Figures 2.5a, b**). Finally, USVs were recorded with a microphone placed 40 cm above the OF floor.

### Analysis of USVs

USVs were monitored with UltraSoundGate Condenser Microphones (CM16; Avisoft Bioacoustics, Berlin, Germany) and recorded with Avisoft Recorder 2.7 software (sampling rate: 214,285 Hz; format: 16 bit). High-resolution spectrograms (frequency resolution:.488 kHz, time resolution:.512 ms) were obtained after a fast Fourier transformation (512 FFT-length, 100% frame, Hamming window, 75% time window overlap), by using the Avisoft SASLabPro 5.2 software. First, USVs were automatically detected using the Avisoft SASLabPro function of “whistle tracking” by adjusting the minimal duration, the hold time, and the peak amplitude. USVs emitted within a frequency range of 19–32 kHz were considered as 22-kHz USVs, and USVs between 33 and 96 kHz were defined as 50-kHz USVs (Brenes et al., 2016). Later, experienced observers manually filtered and selected the genuine USVs based on our own criteria reported elsewhere (Brenes and Schwarting, 2015; Brenes et al., 2016). Briefly, if two 50-kHz elements were at least .048 s apart, two independent 50-kHz calls were counted. A flat call was scored when peak-frequency changes within a single call element were equal to, or lower than 5 kHz. Any change in peak-frequency higher than 5 kHz either within a single 50-kHz element (e.g., the zigzag shape in trills calls) or between two or more overlapped 50-kHz USV elements (e.g., as in all step-calls) was considered as a modulation in peak frequency (FM). Accordingly, the following 50-kHz calls subtypes were measured: 1) flats, 2) step-flats (all elements are flat with at least one overlapped element), 3) trills (one single element), and 4) step-trills (at least one element is a trill overlapped with one or more elements). As the rate of USVs is very variable between animals, the minute with the highest number of calls per animal was selected for USVs classification.

### Gene Expression Analysis

Euthanasia was carried out by decapitation and brains were dissected on ice. The nucleus accumbens, the dorsal striatum, and the hippocampus were collected and prepared as previously reported (Sequeira-Cordero et al., 2013; Rojas-Carvajal et al., 2019). Oligonucleotides for BDNF, TrkB, and CREB were designed elsewhere (Rage et al., 2007; Liu et al., 2010), whereas primers for p250GAP and dnmt3a (p250GAP-F 5′-ATGGATTTCAGGTGGGACTCTTC-3′, p250GAP-R 5′-GCTTTGTTGGGCGAGACTTCAT-3′; dnmt3a-F 5′-AGTCATCCGCCACCTCTTCG-3′, dnmt3a-R 5′-TCTCTCCGTCCTCTCGTTCTTG-3′) were designed using the online tools Primer3 (http://bioinfo.ut.ee/primer3-0.4.0/), Primer-BLAST (https://www.ncbi.nlm.nih.gov/tools/primer-blast/) and OligoAnalyzer (https://www.idtdna.com/pages/tools/oligoanalyzer). Conditions for real-time reverse transcription-quantitative polymerase chain reaction (RT-qPCR) were validated in a Rotor-Gene Q (QIAgen, Germany) according to published criteria (Raymaekers et al., 2009). Relative gene expression was determined by the comparative method with hypoxanthine phosphoribosyltransferase 1 (HPRT1) as a reference gene, which has been widely validated and used for the study of gene expression in rat brain tissues after several experimental conditions (Bonefeld et al., 2008; Santos and Duarte, 2008; Julian et al., 2014; Chapman and Waldenström, 2015; Sequeira-Cordero et al., 2019). In our hands, the use of other reference genes has been discouraged (e.g., actin or glyceraldehyde-3-phosphate dehydrogenase, GAPH) as they can be modified by the housing conditions (unpublished results). PCR reactions contained 4 µl of 1:15 diluted cDNA, 5 µl 2× Syber green (Fermentas, USA), and a final primer concentration of 75 nM for HPRT1, CREB, and p250GAP, and 150, 300, and 200 nM for BDNF, TrkB, and DNMT3A, respectively; in a final volume of 10 µl. After an initial denaturation step at 95°C for 10 min, amplification was performed with 40 cycles of denaturation at 95°C for 30 s, 45-s annealing at 58°C for HPRT1 and TrkB, 63°C for p250GAP, and 64°C for BDNF, CREB, and DNMT3A, respectively; with an extension step at 72°C for 30 s. Additionally, a melting curve analysis (95°C for 15 s, 60°C for 60 s, and 95°C for 15 s) was performed in order to confirm the specificity and primer dimmer absence. Samples were run in duplicates, and the mean values were used for further calculations. Each gene was run individually according to the sample maximization method (Hellemans et al., 2007), with each run including all housing groups. Non-template controls and minus RT controls were also included in order to exclude the possibility of genomic DNA contamination. The threshold cycle (Ct) was calculated using the Rotor-Gene Q Series Software (QIAgen, Germany). mRNA levels were reported both as 2^−ΔCt^ and as normalized values centered around the SH5 group mean (i.e., 100%) expressed in percentages (see **Figure 8**).

### Statistical Analysis

All the analyses were done with IBM SPSS v21 software (IBM, USA). Data were expressed as mean ± standard error of the mean (SEM). The parameters measured in the EE cage were the following: locomotor activity (running, galloping, jumping, and climbing); cage exploration (stretch-attempt posture and sniffing); material/items remodeling (digging, gnawing/chewing, material accumulation, material ripping, and item moving); eating; foraging; social interaction (rough-and-tumble play and chasing); and USVs. When two or more behaviors belonged to one category, they were summed up to be compared with each other. These variables were analyzed using a four-way analysis of variance (ANOVA) with behavior (the different categories), housing (i.e., CEE and REE), minutes (i.e., 1–10), and weeks (i.e., 1–5) as factors. In the OF, locomotion (distance traveled), rearing frequency, grooming duration (total and its subtypes), and USVs (total number and its subtypes) were analyzed with mixed multivariate ANOVAs with groups (i.e., SH2, SH5, CEE, and REE) and days (i.e., 1–4) as between-subject factors and minutes (i.e., 1–15) as a within-subjects factor. When both SH and EE groups were quite similar between each other, a main effect of housing (i.e., SH vs. EE) was estimated with one-way ANOVA. The percentage of USVs subtypes was analyzed within each group with one-way ANOVA with call subtype (i.e., flat, step-flats, trills, and step-trills) as a within-subjects factor. Protected, Fisher's Least Significant Difference (LSD) *post hoc* test was used for multiple comparisons among groups. Bonferroni's adjustment was applied for multiple comparisons among minutes and days, when appropriate. Results of the gene expression were analyzed with one-way ANOVA with groups (i.e., SH5, CEE, and REE) as the between-subject factor followed by controlled, planned contrasts. For all analyses, the effect size was estimated with the partial eta-squared (ƞ^2^_p_) coefficient and the statistical significance was defined as *P* < .05.

## Results

### Experiment 1

#### REE Increases the Activity and the Rate of Appetitive USVs in the Cage

Several lines of evidence have shown that restricted or unpredictable access to rewarding stimuli (e.g., food or drugs of abuse) increases both incentive motivation attributed to reward-predicting cues and approaching and consummatory responses toward the reward (Anselme et al., 2013; Brenes and Schwarting, 2014; Schultz, 2016; Kreisler et al., 2018). Considering that laboratory rodents prefer larger and complex cages, social contact, and exercise (Olsson and Dahlborn, 2002; Van Loo et al., 2003; Heyse et al., 2015), we assume that EE is rewarding for rodents. Rats emit high-frequency (e.g., 50-kHz) USVs in social (e.g., mating and rough-and-tumble play) and non-social rewarding situations (e.g., brain stimulation of reward centers and administration of psychostimulants) (Burgdorf et al., 2000; Williams and Undieh, 2010; Pereira et al., 2014; Brenes and Schwarting, 2015). Out of the different 50-kHz calls, the FM subtypes (e.g., step-flats, step-trills, and trills) are indicative of a high, positive affective state (Burgdorf et al., 2007; Burgdorf et al., 2008; Burgdorf et al., 2011). Thus, we hypothesized that unpredictable, restricted access to EE would intensify the incentive value of the EE cage, increasing exploratory activity and 50-kHz calls during the first minutes of EE exposure. To test this hypothesis, we monitored the behavioral and USVs responses displayed by CEE and REE animals within the EE cage throughout the housing weeks. We found that physical activity and cage exploration (i.e., sniffing, rearing, and stretch-attend posture) were the most frequent behaviors during the whole EE period (behaviors: *F*_(2.15,1285.05)_ = 1653.53, *p* =.001, ƞ^2^_p_ =.74; **Figure 3G**). Both EE groups progressively increased locomotor activity across minutes and weeks, but REE animals did it to a greater extent (groups * minutes * weeks: *F*_(36,500)_ = 3.44, *p* =.001, ƞ^2^_p_ =.20) (**Figure 3A**). Cage exploration decreased over minutes only in REE rats (groups * minutes: *F*_(9,500)_ = 3.72, *p* =.001, ƞ^2^_p_ =.06), but progressively increased over weeks in both EE groups, especially in CEE animals (groups * weeks: *F*_(4,500)_ = 15.60, *p* =.001, ƞ^2^_p_ =.11) (**Figure 3B**). Remodeling and modifying the materials and items of the EE cage was one of the behaviors in which the group differences were the greatest, with such activity being increasingly higher in REE rats (groups * minutes * weeks: *F*_(36,500)_ = 3.44, *p* =.001, ƞ^2^_p_ =.20) (**Figure 3C**). The frequency of foraging (groups * minutes * weeks: *F*_(36,500)_ = 2.27, *p* =.001, ƞ^2^_p_ =.14) (**Figure 3D**) and eating (group * minutes * weeks: *F*_(36,500)_ = 3.94, *p* =.001, ƞ^2^_p_ =.22) (**Figure 3E**) was very low during the evaluation period. These behaviors increased slightly in both groups and, in the case of eating, it was significantly higher in CEE rats. Social interaction increased per minute and over weeks, but only in REE rats (**Figure 3F**). The CEE animals, in contrast, showed irregular frequencies per minute with an inverted U-shaped pattern when analyzed through the weeks (groups * minutes * weeks: *F*_(36,500)_ = 1.70, *p* =.01, ƞ^2^_p_ =.11). Once the animals entered the EE cage, the rate of USVs started to increase progressively in both conditions (minutes: *F*_(9,99)_ = 2.143, *p* =.05, ƞ^2^_p_ =.19) (**Figure 4A**, right panel). When comparing by groups, the total number of 50-kHz calls was higher in REE rats (groups: *F*_(1,99)_ = 89.075, *p* =.0001, ƞ^2^_p_ =.50) (**Figure 4A**, left panel). Over weeks, the rate of USVs showed an inverted U-shaped pattern, which peaked at week two and then decreased linearly in the following weeks (weeks: *F*_(4,99)_ = 15.790, *p* =.0001, ƞ^2^_p_ =.41), with the REE rats showing a consistently higher call rate throughout the housing period (groups * weeks: *F*_(4,99)_ = 6.070, *p* =.0001, ƞ^2^_p_ =.21) (**Figure 4A**, middle panel). When analyzing the USVs subtypes, REE rats emitted more FM calls, especially the subtypes with higher peak modulations (i.e., trills and step-trills) (**Figure 4B**).

**Figure 3:** Behavioral kinetics in the environmental enrichment cage. Physical activity **(A)**, cage exploration **(B)**, material/items remodeling **(C)**, foraging **(D)**, eating **(E)**, and social interaction **(F)** displayed over minutes (left panels) and weeks (right panels). Cumulative average activity **(G)**. Data correspond to frequencies expressed as mean ± SEM. CEE, continuous environmental enrichment; REE,restricted and unpredictable environmental enrichment. Single, pairwise-comparisons between groups: *p < .05; **p < .01; ***p < .001. Comparison between behaviors: ^+++^ *p* < .001.

**Figure 4:** Kinetics of ultrasonic vocalizations in the environmental enrichment cage. Total number of 50-kHz calls **(A)** over minutes (left panel), weeks (middle panel), and its cumulative average (right panel). Fifty-kHz calls' subtypes **(B)** and their respective exemplary sonograms. **(C)** Data correspond to frequencies **(A)** and percentages **(B)** expressed as mean ± SEM. CEE, continuous environmental enrichment; REE, restricted and unpredictable environmental enrichment. Single, pairwise-comparisons between groups: ***p < .001.

To our knowledge, this is the first study describing the kinetics in overt behavior and USVs within the EE cage. This study also provides the first empirical evidence that the motivation to “get environmentally enriched” can be increased by restricting access to the cage unpredictably. Based on the behavioral data, it seemed that REE rats tried to make the most out of their limited time in the cage, which in turn changed progressively the type and the combination of activities they chose to do. During these 10 min, REE rats spent their time traveling around and interacting actively with the cage, the materials, and other rats (**Figures 3A, C, F**). A similar study also found that, as compared to SH rats, EE counterparts displayed higher levels of social and non-social activity within the cage, with the level of such activities being even higher in the group enriched with natural items than in the group enriched with artificial ones (Lambert et al., 2016). As our protocol was designed to enhance the interaction with natural, ethologically relevant stimuli and social partners in a sufficiently large space, the distribution and selection of activities made by the REE rats may shed light on which ethological needs are more urgent to be fulfilled when time is limited. The low levels of eating behavior in REE rats could be the result of the competing motivation to perform different behaviors in addition to the net effect of exercise on appetite, which is known to reduce food intake throughout the regulation of several neural messengers, such as insulin, ghrelin, and the corticotropin-release factor (Kawaguchi et al., 2005; Ebal et al., 2007). Based on the level of activity and USVs displayed in the cage, it can be concluded that such an environment was highly rewarding for all animals, but to a greater extent for those with restrict and unpredictable access to the cage. For instance, the between-group differences in the number of 50-kHz calls were 2.28 and 3.67-fold higher in the REE group, with the lowest call rate of the REE rats being even higher than the highest point of the CEE rats. Considering that 50-kHz calls may signal a state of appetitive incentive motivation (Brenes and Schwarting, 2014; Brenes and Schwarting, 2015), the differences in USVs suggest that unpredictable and restricted access to the EE cage could have extended and enhanced the rewarding properties of the EE stimuli. In support to the latter, we have previously found that rats trained to run a runway to enter a locked running wheel, displayed almost the same latencies and rates of 50-kHz calls than those with the unlocked wheel, suggesting that the structural features of the wheels were equally attractive for both groups (Heyse et al., 2015). Once the rats with the unlocked wheel exercised, the rate of 50-kHz calls increased substantially, indicating that the activity on its own was also rewarding for them (Heyse et al., 2015). As the REE rats were housed in groups of five during the non-EE period, entering the EE cage offered the opportunity for interacting with non-cagemates rats, which could have also been a great source of reward. The higher call rate and the larger percentage of FM USVs seen in REE rats may have resulted from social interactions perceived as more appetitive, although the level of social contact was similar between groups during the first weeks. In fact, rough-and-tumble play and social contact are known to elicit high rates of 50-kHz calls, especially in juveniles (Knutson et al., 1998; Burgdorf et al., 2008). As the call rate increased until week two and then decreased in the following weeks (**Figure 4A**, middle panel), we might suppose that the hedonic and motivational properties associated with novelty, exercise, and social interaction required 2 weeks to reach the highest level. Afterward, the affective response to the EE cage seemed to decrease in all animals, despite the efforts made to maintain the novelty and complexity of such an environment. Complementarily, the reduction in call rate seen on weeks three and four may be associated with an age-dependent effect on social interaction-induced 50-kHz calls. Time spent interacting with conspecifics is known to reduce with age, as well as the emission of and the behavioral response to 50-kHz calls (Salchner et al., 2004; for review, see Seffer et al., 2014). Therefore, the call rate may have reduced, as animals were moving away from the age where rough-and-tumble play is highly frequent (Burgdorf et al., 2008; Seffer et al., 2014). Based on our results, it is unlikely that the changes on USVs constitute a mere byproduct of other behavioral activities. The analysis of USVs provided meaningful insights about the subjective motivational and emotional states of the rat in response to the EE, which might not be otherwise obtained.

#### REE Equals the CEE-Induced Enhancements in Novelty Habituation

We have found that restricted the unpredictable access to EE increased the interaction with social and non-social stimuli and the affective responses to them. Thus, we wondered whether such a more intense and motivated EE experience could translate into a noticeable behavioral outcome. Because the decline of locomotion and rearing in the OF is one of the most consistent, robust, and well-replicated findings of EE in rats (Elliott and Grunberg, 2005; Brenes Sáenz et al., 2006; Brenes et al., 2008; Brenes et al., 2009; Turner and Burne, 2014; Urakawa et al., 2014; Brenes et al., 2016; Rojas-Carvajal et al., 2018; Sampedro-Piquero et al., 2018), we used this paradigm as a behavioral readout of the effects of our housing conditions. As expected, all animals habituated to the OF as noted by the reduction of locomotion (minutes: *F*_(10.87,1827.37)_ = 253.17, *p* =.0001, ƞ^2^_p_ =.60; minutes * days: *F*_(32.63,1827.37)_ = 2.47, *p* =.0001, ƞ^2^_p_ =.04) (**Figure 5A**) and rearing frequency (minutes: *F*_(11.67,1960.63)_ = 61.72, *p* =.0001, ƞ^2^_p_ =.27; minutes * days: *F*_(35.01,1960.63)_ = 2.08, *p* =.0001, ƞ^2^_p_ =.04) (**Figure 5B**) throughout the minutes and days. A detailed analysis revealed that such a reduction on OF activity occurred only in the EE groups, especially after the OF2 for locomotion (minutes * groups: *F*_(32.63,1827.37)_ = 2.37, *p* =.0001, ƞ^2^_p_ =.04; minutes * days * groups: *F*_(97.90,1827.37)_ = 1.43, *p* =.002, ƞ^2^_p_ =.07), and the OF3 for rearing (minutes * groups: *F*_(35.01,1960.63)_ = 2.08, *p* =.0001, ƞ^2^_p_ =.04; minutes * days * groups: *F*_(105.03,1960.63)_ = 1.37, *p* =.009, ƞ^2^_p_ =.07). When comparing locomotor activity between the housing conditions, we found that animals in both EE conditions traveled less distance than their SH counterparts on days 2 to 4 (housing: all *p*-values < .001, ƞ^2^_p_ =.35–.49; LSD: *p* < .05) (**Figure 5A**, middle panel). In addition, SH5 rats traveled more distance than SH2 animals on days 2 and 4 (all *p*-values < .05; LSD: *p* < .05), with the SH5 group also differing from each EE group on all testing days (all *p*-values < .05). Consequently, the cumulative distance traveled was lower in both EE groups than in both SH groups and also the SH2 and SH5 groups differed from each other (groups: *F*_(3,180)_ = 29.621, *p* =.0001, ƞ^2^_p_ =.33) (**Figure 5A**, left panel). When analyzing rearing, both EE groups showed the lowest levels throughout the testing period (housing: all *p*-values < .001, ƞ^2^_p_ =.13–.49; LSD: *p* < .05), but single-group differences were only observed on OF4, where each SH group differed from each EE group (LSD: *p* < .05) (**Figure 5B**, middle panel). The cumulative rearing frequency was lower in both EE groups than in both SH groups with no further differences between the SH and EE groups (groups: *F*_(3,180)_ = 12.319, *p* =.0001, ƞ^2^_p_ =.17) (**Figure 5B**, right panel).

**Figure 5:** Behavioral kinetics in the open-field test. Locomotion **(A)** and rearing **(B)** over minutes (left panel), days (middle panel), and their cumulative averages (right panel). Data correspond to meters **(A)** and frequency **(B)** expressed as mean ± SEM. SH2: Standard housing with two rats. SH5, standard housing with five rats. CEE: Continuous environmental enrichment; REE, restricted and unpredictable environmental enrichment. Single, pairwise-comparisons between groups, CEE and REE vs. SH2 and SH5: *p < .05; ***p < .001; SH2 vs. SH5: ^#^ *p* < .05; ^###^ *p* < .001; and SH5 vs. CEE and REE: ^++^ *p* < .01.

The OF behavior of both EE groups was almost identical, suggesting that being enriched only 50% of the total period did not compromise the effects of EE in this test. Evidence from short and restricted EE protocols have revealed neurobehavioral improvements with 3 h/day over 3 weeks (Stein et al., 2016), 2 h/day for 30 days (Widman and Rosellini, 1990), and 2 h/day for 40 days (Widman et al., 1992), suggesting that partial EE is sufficient to induce the expected reduction of locomotion and rearing in the OF (i.e., enhanced novelty habituation). Alternatively, the restricted and unpredictable access to the cage may have potentiated the stimulating effects of EE compensating the 50% of the time they were not in the EE cage. The EE-induced improvements of non-associative learning agree with previous evidence obtained in the OF (Elliott and Grunberg, 2005; Brenes Sáenz et al., 2006; Brenes et al., 2008; Brenes et al., 2009; Brenes et al., 2016; Rojas-Carvajal et al., 2018; Sampedro-Piquero et al., 2018; Mora-Gallegos and Fornaguera, 2019) and with findings of improved performance in episodic and spatial memory tasks (Sampedro-Piquero et al., 2013; Turner and Burne, 2014; Mora-Gallegos et al., 2015; Brenes et al., 2016; Mármol et al., 2017). From a cognitive perspective, it is interpreted that the faster the decline of the activity, the faster the processing of novel and threatening stimuli (Kempermann et al., 2002; Hughes and Collins, 2010). From an emotional perspective, it is assumed that EE animals become less responsive to mild stressors, as EE typically produces a faster reduction in exploratory and defensive responses in anxiety and fear paradigms (Hendriksen et al., 2010; Mitra and Sapolsky, 2012; Ashokan et al., 2016; Koe et al., 2016). Integrating both perspectives, EE is thought to facilitate the extraction of information about the likely sources of threats during the first testing minutes, which is sufficient to reduce arousal and defensiveness within the test. With repeated exposures, this learning generalizes to the same or similar contexts (Rojas-Carvajal et al., 2018; Rojas-Carvajal and Brenes, submitted). As expected, between-days habituation was currently observed in our EE rats (**Figure 5**). In SH rats, however, no such an effect was detected for locomotion, and in the case of rearing, only a small reduction was observed from OF1 to OF2. We attributed this lack of effects on the handling procedure employed in this experiment. The SH rats were handled more frequently than usual to equate the manipulation received by the EE groups, as they were put in and out of the EE cage several times per week. Therefore, handling may have reduced the behavioral reactivity to the OF until a point where no further reductions were possible. In agreement with our results, lengthy handling procedures (1–6 weeks) have been found to reduce locomotor responsiveness to the OF (Hirsjärvi and Väliaho, 1995; Schmitt and Hiemke, 1998; Costa et al., 2012). In unhandled rats, we have observed a more pronounced activity decay in non-EE rats tested exactly as in this experiment (i.e., on four consecutive 15-min tests) (Rojas-Carvajal et al., 2018), with the levels of locomotion and rearing being ~20% and ~10% higher than those reported here, respectively. Finally, it is worth mentioning that the SH groups differed to each other on locomotor activity, with the SH5 group traveling more distance than the SH2 group (**Figure 5A**). We have initially expected that the social enrichment provided by the SH5 housing would reduce or at least equate the behavioral reactivity of SH2 rats. However, we found quite the opposite. We attribute this effect to the mild stress provoked by cage overcrowding. Over time, the cage area became proportionally smaller relative to the animal size, something that may have occurred to a lesser extent in the SH2 group. We have found the same results in the OF when comparing rats housed in groups of six or pairs (Brenes et al., 2016).

#### EE Differentially Affects Grooming Subtypes and Kinetics in the OF

Besides locomotion and rearing, grooming is one of the most responsive OF parameters to EE. In consequence, it constitutes a suitable candidate for the analysis of particular differences induced by our EE protocols. Regarding its association with stress, two seemingly opposite interpretations have been proposed: 1) grooming is a direct marker of distress emitted as a byproduct of other defensive behaviors; or 2) grooming is a stress-coping response that facilitates emotional de-arousal (Spruijt et al., 1992; van Erp et al., 1994; Brenes et al., 2009; Kalueff et al., 2016; Estanislau et al., 2019). However, the analysis of grooming structure and time course has revealed that both interpretations correspond to different phases of the same behavioral process (Brenes et al., 2009; Kalueff et al., 2016; Rojas-Carvajal et al., 2018; Estanislau et al., 2019; Rojas-Carvajal and Brenes, submitted). To integrate these perspectives, we have proposed that bursts of short cephalic grooming are more likely associated with arousal and distress since they appear at the beginning of tests and then decrease progressively along with exploration and risk-assessment. In contrast, longer and more complex grooming sequences should be part of a de-arousal inhibition system restoring emotional homeostasis, as they increase when habituation is taking place and defensive behaviors are less prominent (Brenes Sáenz et al., 2006; Brenes et al., 2009; Rojas-Carvajal et al., 2018; Rojas-Carvajal and Brenes, submitted). Based on this evidence, we analyzed the structure and kinetics of grooming. Regarding the total grooming time, we found that both EE groups showed the highest scores (groups: *F*_(3,992)_ = 42.03, *p* =.0001, ƞ^2^_p_ =.11) (**Figure 6A**). A detailed analysis of its structure revealed differences between the subtypes (subtypes: *F*_(5,992)_ = 279.77, *p* =.0001, ƞ^2^_p_ =.59), which also varied between groups (subtypes * groups: *F*_(15,992)_ = 44.32, *p* =.0001, ƞ^2^_p_ =.40). Such an interaction between subtypes and groups remained throughout the minutes (subtypes * groups * minutes: *F*_(210,13888)_ = 2.44, *p* =.0001, ƞ^2^_p_ =.04) and days (subtypes * groups * minutes * days: *F*_(630,13888)_ = 1.27, *p* =.0001, ƞ^2^_p_ =.06). Among the different subtypes, cephalic grooming and sequential grooming with variations were the most responsive subtypes to the effects of housing (groups: *F*_(3,180)_ = 58.17, *p* =.0001, ƞ^2^_p_ =.51), following quite the opposite kinetics within the SH and the EE groups (**Figures 6B, C**). On one hand, all animals showed high but irregular levels of cephalic grooming (e.g., in OF1), which decreased throughout the minutes (minutes: *F*_(15,180)_ = 2.46, *p* =.003, ƞ^2^_p_ =.18) and days (days: *F*_(3,120)_ = 6.61, *p* =.001, ƞ^2^_p_ =.14) (**Figure 6B**, left and middle panel). In SH rats, cephalic grooming reduced linearly from OF1 to OF4, whereas in EE counterparts, it abruptly declined from OF1 to OF2 and then remained unchanged thereafter (**Figure 6B**, middle panel). When compared by groups, it was found that EE groups showed less cephalic grooming than both SH groups in OF2, and the SH2 group in OF4 (all *p*-values *p* < .05, ƞ^2^_p_ =.18–.24; LSD: *p* < .05). In consequence, SH groups had the highest levels of cephalic grooming throughout the days (groups: *F*_(3,180)_ = 7.19, *p* =.0001, ƞ^2^_p_ =.12; LSD: *p* < .05) (**Figure 6A**, right panel). On the other hand, sequential grooming with variations increased gradually over minutes (minutes: *F*_(15,180)_ = 15.71, *p* =.0001, ƞ^2^_p_ =.59) and days (days: *F*_(3,120)_ = 11.96, *p* =.0001, ƞ^2^_p_ =.18). A detail inspection revealed that such an effect occurred exclusively in both EE groups, which showed a linear increase throughout the days (minutes * groups: *F*_(21.58,__1193.93)_ = 2.27, *p* =.001, ƞ^2^_p_ =.04; days * groups: *F*_(9,120)_ = 3.24, *p* =.001, ƞ^2^_p_ =.15) (**Figure 6C**, left and middle panel). In OF1, the CEE group showed higher levels of sequential grooming with variations than the other groups (LSD: *p* < .01), being the first OF parameter in which the EE groups differed from each other (**Figure 6C**, middle panel). On the following days, however, such differences were no longer observed as grooming increased gradually in REE rats until reaching the levels of that in CEE counterparts. Consequently, both CEE and REE groups differed from both SH groups from OF2 to OF4 (all *p*-values *p* < .0001, ƞ^2^_p_ =.50–.65; LSD: *p* < .05). The SH5 rats had descriptively higher levels of sequential grooming with variations than SH2 rats, which were marginal on OF3 and OF4. When comparing among groups the cumulative time spent on this subtype, the same pattern was observed: each EE group differing from each SH group (groups: *F*_(3,178)_ = 44.97, *p* =.0001, ƞ^2^_p_ =.43; LSD: *p* < .05) (**Figure 6C**, right panel).

**Figure 6:** Grooming kinetics and subtypes in the open-field test. Total grooming **(A)**, cephalic grooming **(B)**, and sequential grooming with variations **(C)** over minutes (left panel), days (middle panel), and their cumulative averages (right panel). Data correspond to seconds expressed as mean ± SEM. SH2: Standard housing with two rats. SH5, standard housing with five rats. CEE, continuous environmental enrichment; REE, restricted and unpredictable environmental enrichment. Symbols correspond to single, pairwise-comparisons between groups. CEE and REE vs. SH2 and SH5: *p < .05; ***p < .001. SH2 vs. CEE and REE: ^&^ *p* < .05; ^&&^ *p* < .01. CEE vs. REE: ^@^ *p* < .05. CEE vs. REE, SH2 and SH5: ^$$^p < .01.

So far, the behavioral changes induced by both EE protocols on traditional OF parameters were alike. The analysis of grooming structure and time course, however, did reveal particular grooming differences between the EE groups. Supporting our interpretations of the grooming subtypes, we found that cephalic grooming was higher at the beginning of the test, declined with repeated testing, and was lower in EE rats. In contrast, sequential grooming with variations gradually increased with repeated exposures being 2- and 3-fold higher in REE and CEE rats than in SH counterparts, respectively. Contrary to locomotion or rearing, the REE rats required repeated OF exposures to show the same grooming levels observed in the CEE rats, suggesting that in this particular domain, the REE protocol did not fully compensate for the reduced time into the EE cage. EE-induced higher levels of grooming have also been observed in other conditioned and unconditioned anxiety tests (Turner and Burne, 2014; Sparling et al., 2018; Mora-Gallegos and Fornaguera, 2019). Because EE resembles the natural habitat of the rat and reduces the stress of captivity (Swaisgood, 2007; Tarou and Bashaw, 2007), it is improbable that the high levels of grooming observed in EE animals constitute a distress or displacement response indicative of negative emotionality. Instead, the exposure of rats to EE seems to promote a behavioral phenotype in which both defensive and non-defensive responses to stress are not only equally present but also highly efficient (Mitra and Sapolsky, 2012; Estanislau et al., 2019). In this line, specific grooming subtypes should confer particular ethological benefits by helping animals to restore emotional homeostasis and to gradually disengage from defensive responses when they are no longer required (Rojas-Carvajal et al., 2018). We are aware that distress and captivity may induce pathological forms of grooming by excess (i.e., nail-biting, barbering, and stereotypies) or defect (e.g., porphyrin accumulation or dirt accumulation in the fur). However, neither of these signs was observed in our EE rats. As grooming abnormalities have increasingly become a key marker in preclinical models of Autism-spectrum disorder (for review, see Bernard et al., 2015; Kalueff et al., 2016; Zhang et al., 2017), Obsessive-compulsive disorder (Hajheidari et al., 2017), Parkinson disease (Paumier et al., 2013), and Huntington's disease (Tartaglione et al., 2016), EE could be used in these models as a treatment to prevent or restore aberrant forms of grooming (Swaisgood, 2007).

#### EE Reduces Total Calling While Shifting the USVs Subtypes in the OF

Spontaneous 50-kHz calls, especially the flat subtypes, are usually emitted when animals are transiently separated from conspecifics and placed alone in a testing context (Wöhr et al., 2008; Natusch and Schwarting, 2010; Brenes and Schwarting, 2014; Brenes et al., 2016). Flat calls appear at high rates at the beginning of the test and decay over time (Wöhr et al., 2008). This type of USVs is thought to serve both an exploratory and communicative function to maintain or (re)establish social contact and to reduce intra-specific aggression (Wöhr et al., 2008; Natusch and Schwarting, 2010; Brenes et al., 2016). FM 50-kHz calls, such as step-flats, trills, and step-trills, occur at a lower rate during exploratory activities, but appear prominently during social (e.g., rough-and-tumble play, mating, social contact) and non-social rewarding situations (e.g., psychostimulants, food, exercise) (Knutson et al., 1998; Burgdorf et al., 2008; for review, see Brudzynski, 2013). Besides its effects on exploration, risk-assessment, and emotional self-regulation, EE is known to modulate the emission of USVs in the OF (Brenes et al., 2016). To test whether our EE protocols affect prosocial communication, we analyzed the total number of USVs and the call profile during the OF sessions. We found that the total number of 50-kHz calls decreased over minutes (minutes: *F*_(6.07,1068.319)_ = 7.12, *p* =.0001, ƞ^2^_p_ =.04) (**Figure 7A**) but increased throughout the testing days (days: *F*_(3,176)_ = 2.89, *p* =.004, ƞ^2^_p_ =.05), especially when comparing OF1 and OF4 (Bonferroni: *p* < .05) (**Figure 7B**, left panel). Although both EE groups showed descriptively lower 50-kHz calls on each OF, the within-groups variability impeded reaching the significance level. On the cumulative number of 50-kHz calls, both EE groups showed lower levels than SH groups (housing: *F*_(1,176)_ = 4.75, *p* =.03, ƞ^2^_p_ =.03) (**Figure 7B**, right panel). The USVs subtypes were expressed in percentages relative to the total number of 50-kHz calls. When analyzing the flat USVs within days, the percentage of flats increased from OF1 to OF4, but only in the EE groups (housing: *F*_(3,72)_ = 2.99, *p* =.04, ƞ^2^_p_ =.11; Bonferroni: *p* < .05) (**Figure 7C**, left panel). When comparing the housing conditions, EE rats showed a higher call rate than the SH counterparts, especially in OF3 and OF4 (housing: all *p*-values < .01, ƞ^2^_p_ =.16–.17). A detailed analysis showed that CEE rats had a higher call rate than SH2 conspecifics on those days (groups: all *p*-values < .05, ƞ^2^_p_ =.18–.20; LSD: *p* < .05). The cumulative percentage of flat calls was higher in the EE groups than in the SH groups (housing: *F*_(1,175)_ = 17.74, *p* =.0001, ƞ^2^_p_ =.09), with the CEE rats emitting more flat calls than the SH2 and SH5 counterparts (groups: *F*_(3,173)_ = 6.76, *p* =.0001, ƞ^2^_p_ =.10) (**Figure 7C**, right panel). Regarding the FM subtypes, the percentage of trills was lower in EE rats than in SH counterparts from OF2 onwards (housing: all *p*-values < .01, ƞ^2^_p_ =.14–.18) (**Figure 7E**, left panel). The single-group analysis revealed that the CEE rats showed fewer trills than SH2 counterparts in OF3 and OF4, while the REE rats emitted fewer trills than the SH2 conspecifics only in OF4 (all *p*-values < .05, ƞ^2^_p_ =.18–.22; LSD: *p* < .05). Consequently, the cumulative percentage of trills was lower in both EE groups (housing: *F*_(1,175)_ = 21.17, *p* =.0001, ƞ^2^_p_ =.11), with the CEE animals emitting fewer trills than both SH2 and SH5 animals and the REE rats also emitting fewer calls than the SH2 counterparts (housing: *F*_(1,173)_ = 8.40, *p* =.0001, ƞ^2^_p_ =.13; LSD: *p* < .05) (**Figure 7E**, right panel). Over days, step-trills reduced from OF1 to OF3 only in EE groups (housing: *F*_(3,72)_ = 2.77, *p* =.048, ƞ^2^_p_ =.10; Bonferroni: *p* < .05) (**Figure 7F**, right panel). When comparing the housing conditions, a significant and marginal reduction in the call rate was noted on OF3 (*p* =.03; ƞ^2^_p_ =.11) and OF4 (*p* =.08), respectively, with no single-group differences detected. For the step-flats, no main effects or interactions were observed (**Figure 7E**). When comparing the subtype distribution within each group, we found that the SH2 rats emitted flat calls and trills in almost the same proportion, with both subtypes being higher than the step-flats and step-trills (*F*_(3,186)_ = 50.82, *p* =.0001, ƞ^2^_p_ =.45; Bonferroni: *p* < .01) (**Figure 7G**). In the SH5 groups, the flat calls were 1.1-fold higher than the trills, with both subtypes differing from the rests (*F*_(3,111)_ = 50.04, *p* =.0001, ƞ^2^_p_ =.58; Bonferroni: *p* < .01). In the REE group, the proportion of flat calls was 2.05-fold higher than the trills, with the percentages of these subtypes being higher than that of the step-flats and step-trills (*F*_(3,111)_ = 69.13, *p* =.0001, ƞ^2^_p_ =.64; Bonferroni: *p* < .01). In the CEE group, the rate of flat calls was 3.48-fold higher than the trills, with both call subtypes differing from the rests (*F*_(3,108)_ = 105.27, *p* =.0001, ƞ^2^_p_ =.75; Bonferroni: *p* < .01).

**Figure 7:** Ultrasonic vocalizations kinetics and subtypes in the open-field test. Total number of 50-kHz calls over minutes **(A)** and days **(B)**. Percentages of flats **(C)**, step-flats **(D)**, trills **(E)**, and step-trills **(F)**. Distribution of 50-kHz calls subtypes within each group **(G)** and their respective exemplary sonograms (lower panel). Data correspond to frequencies **(A, B)** and percentages **(C–G)** expressed as mean ± SEM. SH2: Standard housing with two rats. SH5, standard housing with five rats. CEE, continuous environmental enrichment; REE, restricted and unpredictable environmental enrichment. Symbols correspond to single, pairwise-comparisons between groups. CEE and REE vs. SH2 and SH5: **p < .001. CEE vs. SH2: ^%^ *p* < .05. CEE vs. SH2 and SH5: ^Ψ^ *p* < .05. REE vs. SH2: ^Δ^ *p* < .05. For pie graphs, see main text for details.

In all groups, the total number of 50-kHz calls reduced during testing minutes but increased throughout OF assessments, with the EE rats showing the lowest rates. This within-test, habituation-like pattern appears after repeated testing and has also been observed in non-EE rats (Wöhr et al., 2008). The lack of differences in call number between the EE groups suggests, again, that partial exposures to EE are enough to produce the effect of full EE or that motivational factors associated with the REE protocol compensated for the less time they were in the EE cage. In any case, EE may have enhanced the information-processing of contextual cues contributing to reducing their social signaling faster than in the SH groups, when recognizing that no USVs feedback from conspecifics or social encounters would occur within the test. The gradual, between-days increase in call rate observed in all animals may have resulted from a reduction in the averseness of the OF as much as habituation was taking place. Animals tested in mild stress contexts, such as an OF with no bedding, usually display low rates of 50-kHz calls (Wöhr et al., 2008; Natusch and Schwarting, 2010), but when they are repeatedly exposed to familiar (i.e., housing cage with bedding) or unfamiliar (i.e., runway maze) contexts, call rate increases progressively over days (Schwarting et al., 2007; Brenes and Schwarting, 2014). In contrast, if animals are exposed to footshock stress, 50-kHz calls are abolished even when testing occurred in a highly familiar context, such as a housing cage filled with fresh bedding (Rojas-Carvajal and Brenes, submitted). When analyzing the call profile, the reduction in total call number observed in the EE groups coincided with a relative increase in flat calls at the expense of the FM subtypes, especially those including trills. In fact, the percentages of flats and FM calls varied proportionally to the level of social EE, with the rats raised in larger groups emitting more flat calls in the OF, in agreement with previous results (Brenes et al., 2016) (**Figure 7G**). As separation-induced flat calls may signal a positive affective state of receptiveness to engage in social interactions and to reduce intraspecific aggression (Wöhr et al., 2008; Brenes et al., 2016), increased social contact during early development seems to favor prosocial competence by optimizing the communicational repertoire according to the particular social demands of the context. Also, the differences in the proportion of flat-to-trills percentages observed between the CEE and REE rats suggest USVs are sufficiently responsive to the degree of stimulation that differentiates both EE groups. An alternative, non-exclusive explanation of the differences in the call profile between groups relates to the level of arousal induced by the OF experience. Novelty and exploration are rewarding for rats and depend on the activity of the mesolimbic catecholaminergic system (Hughes, 1968; Robinet et al., 1998; for review see Bevins, 2001), with dopamine and especially noradrenaline as the main modulators of the stress and arousal responses (for review, see Godoy et al., 2018). FM calls are also highly dependent on that neurochemical system (for a review, see Simola and Brudzynski, 2018), with noradrenaline activity being critical for psychostimulants to increase FM calls (Wright et al., 2012). Thus, the high percentage of FM USVs seen in the SH2 rats may reflect a state of arousal induced by the challenging experience of the OF. In the EE rats, on the contrary, the OF environment was perceived as less novel and exciting in relation to the complexity of the EE cage, which in turn reduced the rate of FM calls. In general, our data showed that the emission of 50-kHz calls was differentially modulated by the degree of EE, both quantitatively and qualitatively.

### Experiment 2

#### REE Alters Gene Expression in the Hippocampus and Dorsal Striatum

EE induces numerous physiological, structural, cellular, synaptic, and molecular adaptations, especially in the hippocampus and the mesocorticolimbic circuits (Bekinschtein et al., 2011; Barros et al., 2019; Ohline and Abraham, 2019). Such adaptations comprise changes in signaling pathways and the expression of several genes underlying the neurobehavioral effects of EE (Simpson and Kelly, 2011; Zhang et al., 2018; Ohline and Abraham, 2019). Thus, we measure the mRNA levels of BDNF, TrkB, CREB, DNMT3A, and p250GAP, based on previous studies and because they are integrated within a signaling pathway related with neural plasticity (Nakazawa et al., 2003; Carlezon et al., 2005; Bayraktar and Kreutz, 2018; Kowiański et al., 2018; Sequeira-Cordero et al., 2019) (**Figure 8F**). In a separate experiment, rats were housed in SH5, CEE, and REE conditions (n=10 animals/group) for 30 days and no behavioral testing was performed. After this period, gene expression analyses were carried out on the hippocampus, dorsal striatum, and nucleus accumbens. In the hippocampus, we found that BDNF was upregulated in the REE group as compared to both CEE and SH groups (*t*_(27)_ = 2.60, *p* =.01, ƞ^2^_p_ =.21), which showed very similar levels (**Figure 8A**). The expression of the TrkB receptor was higher in REE group compared with the CEE group (*t*_(27)_ = 1.78, *p* =.05, ƞ^2^_p_ =.17), with no other between-group differences detected (**Figure 8B**). CREB expression was downregulated in the REE group as compared to both CEE and SH groups (*t*_(27)_ = 2.63, *p* =.01, ƞ^2^_p_ =.29) (**Figure 8C**). In dorsal striatum, both EE groups showed higher BDNF mRNA levels than the SH group (*t*_(27)_ = 2.63, *p* =.01, ƞ^2^_p_ =.29), with the REE group having also higher BDNF expression than CEE group (*t*_(27)_ = −1.99, *p* =.05, ƞ^2^_p_ =.24) (**Figure 8D**). The expression of the DNMT3A was higher in both EE groups compared to the SH group (*t*_(26.67)_ = 2.63, *p* =.05, ƞ^2^_p_ =.10) (**Figure 8E**). No significant differences were observed in the nucleus accumbens.

**Figure 8:** Effects of environmental enrichment on gene expression. Relative mRNA expression of BDNF **(A)**, TrkB **(B)** and CREB **(C)** in the hippocampus, and BDNF **(D)** and DNMT3A **(E)** in the dorsal striatum. The mRNA expression levels in all the brain regions analyzed **(F)**. Data correspond to percentages relative to the mean of the SH5 group **(A–E)** or 2^−dCT^ values **(F)** expressed as mean ± SEM. SH5, standard housing with five rats. CEE, continuous environmental enrichment; REE, restricted and unpredictable environmental enrichment. Symbols correspond to single, planned comparisons between groups. REE vs. CEE and SH5: ^ΘΘ^ *p* < .01. REE vs. CEE: ^@^ *p* < .05. CEE and REE vs. SH5: **p < .01.

Experiment 2 aimed to analyze the effects of our EE protocols on the expression of genes involved in neural plasticity and epigenetic regulation in the nucleus accumbens, dorsal striatum, and hippocampus. Although the nucleus accumbens is well-known to participate in the attribution of incentive salience to reward-predicting cues and appetitive associate learning (Williams and Undieh, 2010; Anselme et al., 2013; Schultz, 2016), no significant differences in gene expression were observed. It is undeniable the nucleus accumbens might have been involved in controlling the motivated responses analyzed in experiment 1, as suggested elsewhere (Burgdorf et al., 2000; Anselme et al., 2013; Schultz, 2016); however, the genes chosen here, the tissue sampling time, and the absence of a behavioral challenge may account for the lack of effects.

Unlike the nucleus accumbens, the hippocampus did show differences in gene expression among groups. For instance, BDNF expression was upregulated only in the REE group, in agreement with one report of intermittent EE (i.e., 12 h per day throughout 7 weeks) (Williamson et al., 2012). Most of the evidence about the upregulation of hippocampal BDNF mRNA or protein comes from studies of continuous EE in rats (Young et al., 1999; Ickes et al., 2000; Williamson et al., 2012; Bechara and Kelly, 2013) and mice (Rossi et al., 2006; Zajac et al., 2010; Kobilo et al., 2011; Kuzumaki et al., 2011; Chourbaji et al., 2012; Tipyasang et al., 2014; Meng et al., 2015). As we found no differences between SH5 and CEE rats, we failed to reproduce such expected results. Variations in the EE protocols, such as cage size, housing density, type and number of items employed, duration of the protocol, age, and species, may account for the discrepancies (for a review see Simpson and Kelly, 2011). Out of these factors, the inclusion/exclusion of running wheels within the EE cage emerges as a critical methodological aspect, since physical exercise (i.e., the use of running wheels or treadmills) is considered the principal stimulus involved in the EE-induced increases in BDNF expression (Zajac et al., 2010; Kobilo et al., 2011; Bechara and Kelly, 2013). Accordingly, many reports describing higher hippocampal BDNF levels included running wheels in their EE protocol (Young et al., 1999; Ickes et al., 2000; Rossi et al., 2006; Kobilo et al., 2011; Kuzumaki et al., 2011; Williamson et al., 2012; Bechara and Kelly, 2013; Tipyasang et al., 2014; Meng et al., 2015), and at least two studies showing no effects or a decrease in BDNF levels did not use this device (Falkenberg et al., 1992; Spires et al., 2004). Although not definitive, this trend supports the role of exercise in modulating hippocampal BDNF expression and may account for the lack of effects in the CEE group, as we did not include running wheels in our protocol. In REE animals, in contrast, the increased physical activity and incentive motivation may have boosted the stimulatory effects of EE on hippocampal BDNF-TrkB expression. Alternatively, as REE animals were enriched only 50% of the time, the upregulation on those genes might have corresponded to an earlier stage of the EE effects, which may have already returned to baseline levels in the CEE group. Nevertheless, the lack of running wheels did not impede finding differences in BDNF expression in the dorsal striatum, pointing out to a region-dependent effect of our EE protocols on neural plasticity. In that region, BDNF expression was upregulated in both EE groups, with the REE group also showing higher levels than the CEE group, indicating that the dorsal striatum is a very responsive region for identifying activity-dependent changes in the brain. Some studies of continuous EE in mice have found similar (Bezard et al., 2003; Tipyasang et al., 2014) or negative results (Spires et al., 2004; Mazzocchi-Jones et al., 2011). Altogether, our findings suggest that, as compared with CEE, REE recruited the BDNF-TrkB signaling to a greater and broader extent. Although brain and behavioral data corresponded to independent experiments, changes in that signaling pathway may have underlain the behavioral improvements seen in the REE group, as it has been shown with protocols of continuous EE (Bekinschtein et al., 2011; Chourbaji et al., 2011; for a review see Barros et al., 2019).

On the other hand, hippocampal CREB expression was lower only in REE rats than in the other groups, with no further differences observed. To our knowledge, there is no evidence of CREB activity after restricted EE. However, the lack of effects in the CEE group disagrees with many reports showing that continuous EE increases CREB mRNA/protein or its phosphorylation in the hippocampus of mice (Huang et al., 2006; Huang et al., 2007; Hu et al., 2013; Du et al., 2017) and rats (Young et al., 1999; Zhang et al., 2016). As one report without running wheels failed to reproduce the EE-induced increases in CREB, this factor could explain the discrepancies (Williams et al., 2001). It must also be considered that many studies showing increases in CREB expression included behavioral testing after the EE protocol (Huang et al., 2006; Huang et al., 2007; Zhang et al., 2016; Du et al., 2017). The exposure to novel contexts, such as testing apparatuses, is known to increase CREB expression and phosphorylation (Moncada and Viola, 2006). As no behavioral testing was included in experiment 2, the interaction between novelty and EE could have been necessary for upregulating the CREB expression in the hippocampus of CEE rats. A similar interaction between behavioral testing and EE has also been reported for hippocampal BDNF expression (Falkenberg et al., 1992). A third alternative explanation should be considered. Biphasic activation of hippocampal CREB has been related to memory formation, with CREB increasing during novelty encoding and decreasing when the stimulus becomes familiar (Moncada and Viola, 2006). Other reports have also found two peaks of CREB activity following associative learning in rats, suggesting that CREB may follow many activational phases (Bernabeu et al., 1997; Stanciu et al., 2001). In our experiment, it is plausible that the putative increase in CREB expression expected for CEE rats had already occurred at an earlier stage and returned to the baseline levels once the EE cage became familiar. In REE rats, this process may have delayed, first because rats remained in the cage only half of the time and second, due to the constant changes and unpredictable access to the cage, which in turn compromised the familiarization to the context. Thus, the reduction in CREB expression seen in the REE group may have corresponded to that stage. As this panorama remains speculative, further research is needed to clarify the functional relevance of these results.

EE increased the expression of DNMT3A in the dorsal striatum. Although the role of DNMT3A as an epigenetic modifier of EE effects has been scarcely studied, at least one report shows an EE-mediated increase of DNMT3A mRNA in the hippocampus of a genetic mouse model of Alzheimer disease (Griñán-Ferré et al., 2018). Furthermore, it is known that EE modulates gene transcription by increasing or decreasing DNA methylation patterns in a locus-specific manner and depending on the brain region (Griñan-Ferré et al., 2016; Zhang et al., 2018). Thus, our results support the point of view that EE, irrespective of being continuous or random, is capable of augmenting the expression of dorsal striatal DNMT3A, which would have resulted in the hypermethylation and transcriptional regulation of particular loci. Presumably, such epigenetic regulation may have been triggered by the increased sensorimotor and social activity and might somewhat explain its plastic neural adaptations, including the upregulation of BDNF signaling in that region. However, given that such epigenetic changes could operate at myriads of genomic locations, additional studies are required to elucidate the physiologic significance of these results.

## Discussion

In this study, we investigated the likely role of motivation in modulating the neurobehavioral effects of EE in rats. To this aim, we modified our EE protocol by including natural stimuli, which were previously screened and classified according to the species-specific behaviors they may elicit. To our knowledge, this is one of the first reports analyzing behavioral kinetics within the EE cage over different time points for 30 days. Also, this is one of the first implementations of a naturalistic EE protocol, and one of the few efforts for describing the protocol in detail, which is a seldom practice in the field leading to replication problems and many inconsistencies within and between labs. Another source of discrepancies is the type of control group used, which varies from social isolation to groups of five or six rats per cage. Here we showed that groups of two or five rats not only differed one another in some parameters but also affected the magnitude at which the significant differences are estimated.

The second and most important implementation of our experiments was the access to the EE cage, which was made restricted and unpredictable in one EE group. We found that the combination of those factors modified the level and type of activities displayed in the EE cage. Although all EE rats were very active and emitted high rates of 50-kHz calls once entering the cage, the large differences between REE and CEE suggest that the rewarding properties of EE were perceived as more pronounced in the REE rats. As physical activity and social interaction decline with time (Salchner et al., 2004; for review, see Seffer et al., 2014), intermittent access to the EE stimuli and cagemates may have prolonged the period in which these activities peak. In consequence, the benefits derived from physical and social stimulation could have extended during a developmental window that is very sensitive to EE (for review, see Simpson and Kelly, 2011). Thus, the increased activity and incentive motivation associated with the EE may account for the neurobehavioral effects of the REE, which equaled or even surpassed those observed in the CEE group, although REE rats were only 50% of the time on EE. We cannot rule out, nevertheless, that for some neurobehavioral parameters, a short EE experience was enough to induce a ceiling effect in which longer EE exposures exerted no further changes. Although the behavioral and brain data were collected on different experiments, it is possible to think that the boost in the BDNF/TrkB signaling induced by REE was responsible for its behavioral performance. Alternatively, it should be considered that each EE protocol produced its effects following different kinetics, especially at the level of gene expression. As CEE rats accumulated in the first two weeks all the stimulation that REE rats received during one month, the effects seen in the REE brains may have been a rightward shift in the peaks of up- or down-regulation in gene expression with their respective behavioral consequences. In the CEE rats, in contrast, all these neurobehavioral dynamics may have diminished or already returned to baseline levels earlier than in REE rats. Further research is warranted to test all these hypotheses experimentally.

Taken together, our results suggest that short but highly rewarding interactions with a stimulating context induce positive effects on brain and behavior, which are comparable or even superior to those produced by a longer period. People living in urban areas spent most of their time working indoors and living in very impoverished environments with little physical and recreational activities during the day (Biernat et al., 2010; Thorp et al., 2012), constituting a lifestyle that has gradually become the “standard housing” of human beings. The reduction of green areas and sports parks in modern cities has jeopardized the engagement on recreational activities and physical exercise (Haaland and van Den Bosch, 2015). At best, some subjects will spend few hours a week on exercise or outdoor activities, with most people having occasional and minimal access to “enriching” environments. In worst-case scenarios where these activities are rather limited and social contact could be even prohibited –as is the case of sanitary emergencies caused by viral outbreaks (e.g., AH1N1, SARS-CoV-2)– the opportunities to “get enriched” could be virtually nil. Therefore, the use of short and restricted access to EE and exercise would serve to model many aspects of modern life and may have greater translational value than protocols of continuous exposure to stimulation, especially because it is almost impossible for humans. In this line, providing restricted but highly attractive interventions including physical and social activities, may cause a significant impact on an individual's health at lower time and economic costs and with higher treatment's adherence and efficacy. Thus, the design of personalized interventions based on individual interests and motivations may be a powerful tool for improving or replacing traditional treatments and interventions, which may function as a sort of adjuvant, endogenous pharmacotherapy for patients (Sale et al., 2014). At a different level, the implementation of more attractive educational and recreational programs taking into account personal needs and expectations would benefit disadvantaged infantile populations with limited access to stimulating socio-educational contexts.

## Data Availability Statement

The datasets generated for this study are available on request to the corresponding author.

## Ethics Statement

The animal study was reviewed and approved by Institutional Committee for Animal Care and Use of the University of Costa Rica (approval number: CICUA-161-16).

## Author Contributions

JB, MR-C, and AS-C conceived and designed the experiments. MR-C and JB conducted the experiments. MR-C and JB designed and contributed to the analysis of the cage kinetics and the grooming classification. MR-C and JB analyzed the raw behavioral data. AS-C performed the gene expression analysis. MR-C and JB did the statistical analyses. All authors wrote and reviewed the manuscript.

## Funding

This research was supported by the projects 837-B7-603 (Neuroscience Research Center), 723-B7-610 (Institute for Psychological Research), and 742-B4-240 (Institute for Health Research), University of Costa Rica. These projects were awarded with the Research Stimulus Fund of the Vice-rectory of Research, University of Costa Rica. We especially thanks to Mónica Sánchez, Brenda Mendez, Fernanda Calderón, David Ramírez and Johanna Akerman for their assistance with this project. We also thank PhD Jaime Fornaguera Trías, technicians, and the administrative personal for their collaboration in this work.

## Conflict of Interest

The authors declare that the research was conducted in the absence of any commercial or financial relationships that could be construed as a potential conflict of interest.
